# Combine performance, draft position and playing position are poor predictors of player career outcomes in the Australian Football League

**DOI:** 10.1371/journal.pone.0234400

**Published:** 2020-06-17

**Authors:** Benjamin J. Gogos, Paul Larkin, Jade A. Z. Haycraft, Neil French Collier, Sam Robertson

**Affiliations:** 1 Institute for Health and Sport (*iHES*), Victoria University, Melbourne, Australia; 2 Maribyrnong Sports Academy, Melbourne, Australia; University of Illinois at Urbana-Champaign, UNITED STATES

## Abstract

Physical testing-based draft combines are undertaken across various sporting codes to inform talent selection. To determine the explanatory power of the Australian football league (AFL) draft combine, participants drafted between 1999–2016 (*n* = 1488) were assessed. Testing performance, draft selection order and playing position, AFL matches played, AFL player ranking points and AFL player rating points were collected as career outcomes. Boosted regression tree analysis revealed that position and draft selection order were the most explanatory variables of career outcomes. Linear modelling based on testing results is able to explain 4% of matches played and 3% of in-game performance measures. Each individual combine test explained <2% of the matches played outcome. Draft selection order demonstrated mixed results for career outcomes relative to playing position. For instance, key forwards and draft selection order were observed as a slight negative relationship using the AFL Player Ranking points career outcome measure. These findings indicate that the AFL draft combine is a poor measure for informing talent selection, thus providing minimal utility for the practices investigated in this study.

## Introduction

In sport, talent identification (TID) refers to the process of recognising participants that are likely to excel in future [1]. Thus, successful TID hinges on the ability to effectively value the explanatory capacity of each aspect informing selection. This has implications for the on-field success of the organisation and subsequent financial effects which may restrain off-field competitiveness (i.e., coaching staff, training facilities). Talent scouts are duly afforded access to resources such as a draft combine (i.e., an anthropometric and physical testing event), to enhance their judgement prospects. However, TID presents challenges due to a range of variables including non-linear development processes [2, 3], non-genetic factors restraining performance (i.e., socio-economic) [4], subconscious biases towards specific skillsets [5] and unstable physical characteristics during maturation [6]. Thus, the unidimensional constructs often assessed in such combines may contribute to poor selection outcomes [7–9]. As such, it is important to establish the explanatory power of draft combine performance for predicting a player’s long-term career success at the elite level.

Forecasting career outcomes through draft combine performance has been undertaken across various sports (e.g. American football, basketball, ice hockey) with mixed results [8, 10–14]. Weak associations between draft combine testing results and career performance have been observed within the National Basketball Association (NBA), National Football League (NFL) and National Hockey League (NHL) [7–10, 12–16]. Importantly, nuance exists within these findings, as certain combine performance variables are strongly associated to specific position types (e.g., running vertical jump and an NFL wide receiver career performance) [7, 8, 13–15]. Whilst combine performance may not relate to career performance outcomes, it has been shown to accurately explain draft selection order, their salary and signing bonus [10].

In Australian football (AF), attempts have been made to determine the utility of the sport’s version of the draft combine. For instance, performance at the AFL draft combine is strongly associated with selection into the elite AFL competition [1, 17–19], though weakly associated with career performance measures (i.e., matches played) that lack in-game performance context. In one example, 75% of players tested with a 20m sprint speed of <2.99s and multistage fitness score of >14.01 were drafted [1]. Combine performance and imprecise career performance measures (i.e., career games played to end of 2003 season, subjective rating for career potential and 5-point scale career value), were found to have small-to-moderate correlations [19]. Notably, combining match performance measures (i.e., in-game sprint count) with combine performance improved career performance prediction models [20]. Whilst previous studies have investigated the relationship between combine and career performance, they have been restricted by the limited career outcome measures available.

Until recent developments in player performance analytics, games played has predominated as the sole measure to objectively inform career outcomes in AF [17–19, 21]. In the absence of in-game performance measures, researchers created subjective performance ratings to explore the draft combine predictive power [19]. The development of player performance models specific to the AFL provide an opportunity to investigate relationships between pre-career metrics and senior career performance [19, 20]. Consequently, Champion Data (Pty, Ltd) introduced the AFL Player Ranking in 2006, and the AFL Player Rating in 2013. The AFL Player Ranking model is derived from over 100 variables, although is yet to be publicly validated [22]. The AFL Player Rating model is based on the principles of field equity and quantifies a player’s actions relative to how they affect their team’s likelihood to score next. In 94.2% of instances, the team which totalled higher rating points, won the match [22]. Therefore, it is now possible to investigate a player’s performance at the AFL draft combine in relation to a player’s career performance and thus informs the aims of this research.

The primary aim of this study was to investigate the explanatory power of the AFL draft combine data on three measures of career performance: i) the number of games played during a player’s career and a player’s average career performance using ii) AFL Player Rating and iii) AFL Player Ranking models. The study also aimed to determine what additional explanatory power is provided in predicting career performance by including draft selection order and their playing position (i.e., midfield, forward, defender).

## Methods

### Sample

The dataset was generated using a retrospective cross-sectional sampling design and includes a period between 1999 and 2016. Combine test data were collected from players attending the Under 18 (U18) AFL National combine (*n* = 918), State combine (*n* = 271) or another type of combine run by AFL teams, academies or other competitions (*n* = 299). The sample was limited to AF players who had finished their careers (i.e., retirement, delisted). From the complete sample (*n* = 1488), 77% played an AFL match (*n* = 1148) and 36% received an AFL Player Ranking and/or AFL Player Rating (*n* = 536).

### Draft combine

All of the physical and anthropometric testing were conducted in accordance with the standardised AFL draft combine testing protocols [21]. The physical fitness assessment items in the AFL draft combine include a 20-m Multi-Stage Fitness Test (MSFT), 20-m sprint, 3-km time trial, AFL sprint recovery, AFL agility test, running vertical jump, standing vertical jump and a Yo-Yo Intermittent Recovery (IR) test. More detailed descriptions of the physical fitness tests are reported in Woods et al; (2015) and Tanner & Gore; (2012) [21, 23]. Anthropometric testing refers to measurements of arm length, hand span, height, mass, sit and reach and skinfolds. Detailed descriptions of anthropometric tests are reported in Young et al; (2005) [24].

All of the physical and anthropometric testing were administered by industry professionals and conducted in accordance with the AFL Draft Combine testing protocols (21). The testing protocols remained unaltered throughout the research period. Due to the longevity of the study, no further action were taken to minimise potential measurement errors.

None of the researchers were involved with the administered combine tests.

### Career performance

Each player was assigned to a playing position (e.g., general defender, general forward, key defender, key forward, midfield, midfield-forward, wing, ruck) based on the official Champion Data classification. A player’s position is classified at the end of their career by Champion Data and is determined by the position on the field where a player played most of their game time. A definition of each player’s role is available in Table 1.

**Table 1:** Champions data’s descriptions of the seven player roles used in this study.

Playing Position	Definition
General Defender	Plays a role on opposition small-medium forwards and usually helps create play from the backline
Key Defender	Plays on opposition key forwards with the primary role of nullifying his opponent
General Forward	Plays predominantly in the forward half of the ground but with more freedom than a key forward
Key Forward	Plays predominantly as a tall marking target in the forward line
Midfielder	Spends the majority of time playing on the ball
Midfield Forward	Splits time equally between the forward line and the midfield. Often lines up on the half-forward flank but plays a significant amount of time in the midfield
Ruck	Has the primary role of competing for hit-outs at a stoppage
Wing	Spends the majority of time playing on the wing

Career performance data were collected from www.afltables.com and Champion Data (Pty Ltd). The career performance data included matches played, AFL player rankings, AFL player ratings and draft selection order. Matches played refers to the number of AFL appearances by the player. The AFL Player Rankings model includes over 100 variables [22] and was popularised by the fantasy competition, Supercoach (www.supercoach.com.au). Based on the principle of field equity, the AFL Player Rating model is determined by the relative effect a player’s action increases or decreases their team’s expected value of the next score [25]. This concept of expected value is based on contextual information relating to each possession of the ball (i.e. pressure from opponents, field position, and time of the match) [22].

#### Draft selection order

The national draft, held annually during November, determines the order in which players are selected for AFL clubs. On average, 76.7 (± 4.4) players have been drafted per year between 2010–2016. Each AFL club is required to make three selections in the national draft. The selection order for each club is, by and large, determined by the finishing order of the previous season’s AFL competition (e.g., team finishes 18^th^ receives 1^st^ draft selection). There are some circumstances when this order is not followed, such when poorly performing clubs are allocated extra selections in a draft [26]. The selection order is also influenced by the trading of draft selections between clubs, alongside the recent innovation to allow clubs to trade future draft selections [26]. Players who were not selected in the national draft, may subsequently be selected in the rookie draft. The rookie draft is a secondary selection period for first year players and is often used as a prospective form of talent selection (i.e., players selected from other sports). On average 56.7 selections (± 13.6) are made during a rookie draft. Players who were selected in the rookie draft are ineligible for AFL unless they are replacing a teammate who has retired during the season or has suffered a long-term injury [27].

For the purposes of this study, draft selection order was determined by the position the player was selected at and which draft they were selected from. For instance, the last player selected in the national draft at pick 90 would correspond to selection position, 90. The first selection in the rookie draft, which proceeds after the national draft, would correspond to selection position 91.

The AFL gave us permission to use the draft data and written ethics approval was granted by the Victoria University Human Research Ethics Committee (HRE19-015).

### Statistical analysis

#### Linear models

All analyses were conducted using R version 3.6.0 [28]. Visualisations were made using the *ggplot2* package [29]. We first visualized the data to better inform model-building. One key visualisation was a matrix scatterplot produced using the *ggpairs* function in the *GGally* package [30]. The response variables for the models investigating career outcomes were: (1) the total games played during a career; (2) a player’s career mean AFL player rating and (3) a player’s mean AFL player ranking. Three models were fitted to each response variable. Each model within a model set used a different set of predictors. The first model in a set used a set of metrics recorded for each player during the AFL Draft Combine which we denote as ‘Combine’. The second model in a set included Combine and the player’s draft position which we denote ‘Selection’. The third model in a set used Combine, Selection and *a prior* playing position of each player which we denote ‘Position’ in the model notation.

The models fitted to the observed AFL player ratings and AFL player rankings assumed that the residual errors of the models’ fitted values were Gaussian distributed and that the samples were independent and identically distributed. The models were fit using the lm() function. The residuals of the fitted models were inspected in order to make a judgement about the adequacy of the model fits. None of the diagnostics and inspections of residuals led us to believe the models were not appropriately fitted to the data.

This study sought to assess linear relationships and this analysis was undertaken using the Pearson correlation coefficient.

#### Bayesian information criterion

The Bayesian Information Criterion (BIC) is a metric used to select the best model from a set of candidate models. The basis of BIC is the maximum likelihood of the data given the model. The maximum likelihood is then penalized based on the sample size and parameters in the model. Models with more predictor variables are therefore penalised more strongly, which helps avoid issues of over-fitting. The model with the lowest BIC value is usually selected as the best model from the candidate set [31]. BIC was used in conjunction with r-squared to assess which was best at fitting to the data and how much variation was explained by the best model.

#### Boosted regression trees

The distribution of the matches played variable was not normally distributed, suggesting a violation of assumptions for linear models (i.e., errors are normally distributed with a mean of zero). A visual inspection of the response variable showed the data contained a large proportion of zeros and were highly dispersed. Furthermore, when the variable was plotted against each of the predictors, the data showed a distinct ‘clumping’ in the middle of the predictor distributions. This evidence suggested linear models would be inappropriate for modelling the total career games played as a function of the predictors. If the clumping was not evident in the data, we could have fit linear models that accounted for the zero inflation and the over dispersion of the response variables (e.g. zero-inflated negative binomial regression). Instead, we chose to fit boosted regression tree models to the data, or sometimes referred to as gradient-boosted machine learning [32].

The boosted regression tree models were built using the gbm.step() function from the *dismo* package [31]. We fitted several models with different parameter combinations in order to make an informed judgement about the final parameter specifications. We fitted the final models using a tree complexity value of five, a learning rate of 0.001, a bag fraction of 0.5 and assuming a Poisson distribution for the residual errors. We plotted the fitted values as a function of the observed values for each model.

## Results

The combine participants had an average age of 18.5 years (± 1.52) of age, 1.87 (± 6.93) m tall, and a body mass of 81.31 (± 7.8) kg. The summary dataset is limited to AF players with ≤ 1 AFL player rating (*n* = 536) (Table 2).

**Table 2:** Summary of dataset.

Position	N	Matches Played	AFL player rating (mean)	AFL player ranking (mean)
Gen Def	130	77.4	7.2	60.3
Gen Fwd	139	63.2	7.2	55.9
Key Def	52	76.5	7.0	56.2
Key Fwd	58	60.8	6.3	54.1
Mid	48	74.5	7.5	60.9
Mid-Fwd	38	77.0	7.3	60.1
Ruck	30	75.7	7.4	62.0
Wing	41	79.0	7.0	62.3

The number of matches played was negatively correlated with draft selection order (r = -0.35 (95% CI: -0.405, -0.29), t = -11.34, df = 919, p < 0.001) (Fig 1). However, the data were positively skewed and displayed a high level of variance. It also contained a large proportion of zeroes which appear to be more common as draft selection order increased.

**Fig 1:** Relationship between draft selection order and matches played.

Fig 2 displays the relationships between all of the AFL Draft Combine metrics and career matches played. All the variables were weakly correlated with career matches played, ranging from -0.0845 to 0.0513. The Yo-Yo Intermittent Recovery (*r* = .0513), the sum of the anthropometric measures (*r* = .0371) and the right leg running vertical jump (*r* = .0112) were the only three tests with statistical support for the correlation being greater than zero.

**Fig 2:** Correlations of anthropometric measures, draft combine performance and matches played.

The draft combine variables explained 3% of the variation in the AFL Player Rating (Table 3). The model which fit the data included Draft combine and Draft selection order predictors. The model explained 4% of the variance in AFL Player Rating. The inclusion of playing position did not improve the fit of the model to the data.

**Table 3:** Summary of model outputs for AFL Player Rating.

Model	Df	logLik	BIC	Deviance	Adj-R2
Null	1	-1150.71	2313.78	3291.84	0.00
Combine	12	-885.25	1847.72	2348.40	0.03
*Draft combine + Draft selection order	13	-831.17	1744.75	2134.20	0.04
Draft combine + Draft selection order + Playing position	20	-826.55	1776.71	2080.13	0.04

The Asterix denotes the best fitting model base on the lowest BIC value.

The Draft combine variables explained between 3% and 6% of the variance in AFL Player Ranking (Table 4). The best fitting model included the draft combine and draft selection order predictor variables and explained 3% of the outcome variance. The inclusion of playing position doubled the percentage of variance explained but reduced the model fit.

**Table 4:** Summary of model outputs for AFL Player Ranking.

Model	Df	logLik	BIC	Deviance	Adj-R2
Null	1	-2622.79	5258.23	383522.20	0.00
Draft combine	12	-2118.07	4315.53	328979.43	0.03
*Draft combine + Draft selection order	13	-2020.63	4126.05	322287.11	0.03
Draft combine + Draft selection order + Playing position	21	-2009.60	4152.44	306058.42	0.06

The Asterix denotes the best fitting model base on the lowest BIC value.

The boosted regression tree scatterplot (Fig 3) demonstrates the capacity to fit career outcome performance (i.e., AFL games played) with each of the three models (i.e., Combine, Combine + Position, Combine + Position + Selection). The figure indicates that improvements in fitted value to career outcome are most apparent when player position and draft selection are combined with combine performance.

**Fig 3:** Boosted regression tree scatterplot of matches played and the fitted values of each model. Combinations of predictor variables as follows; combine, combine + playing position, combine + playing position + draft selection order.

Fig 4 shows the relative importance of each predictor variable for each of the three boosted regression models. The agility test and the skinfold test were near equally important predictors for the model that included only the draft combine predictors. No predictor had an importance value greater than 15%. Player position was by far the most important predictor variable in the model that used the draft combine data and playing position data. Playing position had a relative importance value greater than 35%. The next most important predictor was the skinfold test at approximately 10% importance. The remaining predictors in this model had a relative importance of less than 10%. The most important predictors of the final model were playing position and draft selection order. Again, playing position had a relative importance value of 37%. Draft selection had a relative importance of more than 25% and the draft combine predictors had relative importance values of less than 10%.

**Fig 4:** Relative influence of the predictor variables based on each of the boosted regression tree models. Combinations of predictor variables as follows; combine, combine + playing position, combine + playing position + draft selection order.

The relationship of draft position and AFL career matches played by field position demonstrates similar findings across positions (Fig 5). The key forward positions has the greater symmetry.

**Fig 5:** Relationship between draft selection order and matches played relative to playing position.

Midfielders, midfield-forwards and rucks demonstrate a positive skew when measuring the relationship between draft position and match performance models (Figs 6 & 7). Wings, general defenders, general forwards and key defenders are normally distributed. Key forwards indicate a slight negative skew in relation to AFL Player Ratings. This finding suggests that key forward AFL Player Rating performance and draft position are unrelated or more successful at a later selection. The AFL Player Rankings demonstrates similar findings, with wingmen and key forward slightly more positively skewed. A symmetrical result reflects a non-causal relationship between draft position and match performance. Successful draft selection from a match performance perspective has been achieved at alternate rates relative to AF player field position.

**Fig 6:** Relationship between draft selection order and AFL Player Rating mean relative to playing position.

**Fig 7:** Relationship between draft selection order and AFL Player Ranking mean relative to playing position.

## Discussion

This study demonstrates the forecasting value of the AFL Draft Combine, across a longitudinal measure (i.e., matches played) and two match performance rating models (i.e., AFL Player Ratings and AFL Player Rankings). Further, the importance of a positional breakdown in talent evaluation is evidenced, as selection outcome varies between positions. Previously, the predictive validity of the AFL Draft Combine on career outcomes has been examined without in-game performance models and thus used subjective based measures (i.e., professional opinion) [19–21]. However, with a validated match performance rating model now available [22], scrutinising career outcomes with increased rigour is viable. Results demonstrated the limited forecasting capacity of the AFL Draft Combine and mixed selection outcome across multiple position types, informing appropriate decision weighting within professional talent selection.

Modelling career outcomes based solely on testing combine profiles, is recognised as a limited endeavour [8, 12, 13, 19, 21]. This study found that combine measures explained less than 3% of the variance in career outcomes for AF players, and less for longevity than match performance. Combining the draft selection order and combine performance improved the longevity model minimally, and the combination explained less or similar career outcomes for the in-game measures. Individual tests were weakly associated with career outcome measures. This may indicate that either the rating model is failing to recognise (e.g., leadership skills) skillsets important for match selection, or that factors unrelated to match performance may be inhibiting match selection [33, 34]. Comparable results have been noted within the NFL, with combine explaining 30% and 24% of the variance across a variety of sport specific outcome measures [8, 12]. Similarly, AF players who performed one standard deviation above the mean for Draft Combine testing results were assessed as a small magnitude of difference [20]. Conversely, NBA findings demonstrate a medium to large correlation between anthropometrics and certain phases of play [13]. This is an uncommon finding and although speculative, may be results of specific elements of the sport (e.g., vertical jump performance and the necessity to compete aerially in basketball), rather than specific combine testing protocols.

A plausible explanation for the lack of association between combine performance and career outcomes is that the tests measure physical fitness characteristics, and are not representative of in-game AF-playing skill and ability. Skill is defined as a narrow focus on a particular task, whilst ability is competency across multiple sets of tasks [35]. For example, a ruckman may have an exceptional vertical jump and yet mistimes the hit out contest, resulting in a negative performance outcome. Thus, vertical jump performance does not necessarily equate to elite ruck performance. AF is a complex sport regardless of position, demanding a multitude of physical, technical and decision making characteristics for successful performance [36]. These findings suggest a task specific model of a draft combine may provide improved explanatory power [20, 37, 38]. An initial investigation revealed combine performance becomes more explanatory when combined with in-game sprint count [20]. Thus, a combine limited by its lack of specificity, will presumably be improperly purposed to relate to a measure accounting for numerous in-game performance indicators.

Draft combine based modelling demonstrate similar explanatory power for in-game career performance measures as they do for longevity markers. Prior to the validation of the AFL Player Ratings metric [22], matches played was the sole objective career outcome measure and thus has been prevalent throughout the AF TID literature [19–21]. Notably, draft combine testing results explained less than 4% of the variation in career matches and 3% for in-game performance measures (Fig 2). Differences are noticeable between the BIC in-game performance rating models, as the BIC performance is noticeably improved for the AFL Player Ratings. Differences in relation to scoring distribution and scoring methodology are probable rationalisations for the findings. As the AFL Player Rating model is informed by the principle of field equity, it may be assessing trends less observable to the human eye, in comparison to the Rankings model (which includes disposal efficiency and contested marking measures). Future research may look to determine the construct validity of the AFL Player Rankings, for comparative purposes.

Differences in selection outcome were recognised between positions, with positive selection more reliable for midfielders and rucks. For general defenders, general forwards, key position defenders and key position forwards, weak relationships were observed between draft selection order and match performance models. A slight negative correlation existed for key forward draft selection order and in-game performance rating models. Thus, draft selection order is unrelated to performance within the key forward position. This may be indicative of the evolution in AF which in modern times is largely characterised by field dominance and coordinated defensive press strategies, prioritising skillsets uncommon in traditional key forward players [39]. It must also be recognised that this may be due in part to the relatively minimal number of key forwards selected (*n* = 58). Alternatively, midfield selection appears successful as early draft order status is related to positive match performance ratings and matches played. However, it remains unclear whether this is due to positive talent selection choices or because successful AF players are more likely to migrate toward the midfield position, characterised by the last 13 Brownlow medallists (i.e., the player voted the competition’s best and fairest player) primarily playing as midfielders [40]. General defenders and general forwards performed similarly across all career outcome measures to key positions, with limited relationship between draft order and match performance ratings. Whilst this may be a result of sub optimal talent selection practices within this positional demographic, there could also be limitations with the models for appropriately adjudicating these positions [22]. Notably, a divergence in results is present for matches played and draft selection order, suggesting a presence of loss aversion bias [33, 34].

Prospect theory refers to loss aversion bias as individuals whom are more sensitive to the possibility of losing value than they are attaining the same value [33, 34]. From a sporting perspective, this applies to early selection and the readiness to select the athlete for performance, with limited regard for the athlete’s performance level. The discrepancy between matches played, AFL Player Rankings and AFL Player Ratings, relative to draft selection order (Figs 5, 6 & 7), indicates that early draft selection is provided more opportunity (i.e., increased matches player) than later selection, irrespective of in-game performance. This finding may signify that decision making (i.e., match selection, contract offers) can be less rational than if bereft of these factors. Future research may seek to explore this possibility across numerous sports.

## Conclusion

The data collected at the AFL draft combine are poor predictors of career performance. Predictors like draft position and playing position provide only small improvements in explanatory power. Notably, midfield-oriented positions (i.e., midfielders, midfield-forwards, rucks) demonstrated a positive relationship between selection order and match performance rating models, whilst all other positions were less clearly defined. Discrepancies between matches played and in-game performance measures relative to selection order may also identify the presence of a loss aversion bias. This research can be used to appropriate confidence levels in measures informing talent selection (i.e., AFL Draft Combine) and identify patterns of selection performance relative to player position.

## Supporting information

S1 Dataset De-identified dataset of all players. (XLSX)
